The article "Risk Assessment of Critical Obstetric Bleeding With Low-Molecular-Weight Heparin" was published in 2024. Journal: Cureus.

# Risk Assessment of Critical Obstetric Bleeding With Low-Molecular-Weight Heparin

**DOI:** 10.7759/cureus.59933

**Published:** 2024-05-08

**Authors:** Miho Akaishi, Kunio Tarasawa, Hirotaka Hamada, Noriyuki Iwama, Hasumi Tomita, Tetsuya Akaishi, Kiyohide Fushimi, Kenji Fujimori, Nobuo Yaegashi, Masatoshi Saito

**Affiliations:** 1 Department of Obstetrics and Gynecology, Tohoku University, Sendai, JPN; 2 Department of Health Administration and Policy, Tohoku University, Sendai, JPN; 3 Department of Education and Support for Regional Medicine, Tohoku University Hospital, Sendai, JPN; 4 Department of Health Policy and Informatics, Tokyo Medical and Dental University, Tokyo, JPN

**Keywords:** obstetrical disseminated intravascular coagulation (dic), unfractionated heparin, low molecular weight heparin, critical obstetric bleeding, anticoagulants

## Abstract

Background: Use of unfractionated heparin (UFH) during the peripartum period is considered to be a higher risk of critical obstetric bleeding compared to low-molecular-weight heparin (LMWH). However, the evidence for the safety of using LMWH during the peripartum period is currently lacking.

Methods: This study retrospectively investigated a nationwide medical database to clarify the safety of using LMWH during childbirth. The Japanese Nationwide Diagnosis Procedure Combination database was retrospectively reviewed, and data from women with childbirth between 2018 and 2022 were collected.

Results: Among the overall 354,299 women with childbirth, 3,099 were with obstetric disseminated intravascular coagulation (DIC), 484 were with critical obstetric bleeding requiring massive red blood cell (RBC) transfusion ≥4,000 cc, and 38 were with maternal death. Among the overall women, each of the anticoagulants other than LMWH was associated with critical obstetrical bleeding with an adjusted odds ratio (aOR) greater than 1.0, while LMWH was not associated with critical obstetrical bleeding (aOR, 0.54 (95% confidence interval, 0.11-2.71)). This finding did not change in subgroup analyses among those with Cesarean section. Furthermore, UFH was associated with critical bleeding among the 3,099 women with obstetrical DIC (aOR, 3.91 (2.83-5.46)), while LMWH was not (aOR, 0.26 (0.03-1.37)).

Conclusion: The use of UFH was significantly associated with an increased critical obstetric hemorrhage requiring massive RBC transfusion or total hysterectomy. Meanwhile, the use of LMWH was not associated with increased critical obstetric bleeding. LMWH would be safer than UFH to be used for women during childbirth.

## Introduction

Critical obstetric bleeding is among the major causes of maternal death during childbirth. As an obstetric condition underlying critical obstetric bleeding, obstetrical disseminated intravascular coagulation (DIC) occurs in 0.03%-0.35% of all pregnancies [1-4]. It is among the common causes of maternal deaths during childbirth, with the maternal mortality rate due to DIC being approximately 1.0% in Japan [5-7], which is considered to be among the lowest worldwide [8]. A previous study from a tertiary medical center in Turkey reported that the mortality rate of obstetric DIC may be as high as 25% [9]. Obstetric DIC triggers excessive consumption of blood coagulation factors and platelets, resulting in critical bleeding and organ dysfunctions due to the co-occurrence of overactive coagulation and fibrinolysis [10,11]. Obstetric DIC is secondarily triggered by various obstetric conditions, such as placental abruption, amniotic embolism, atonic bleeding, and retained stillbirth [12-16]. It is an emergent condition, with most maternal deaths reportedly occurring within 24 h of childbirth [17]. Early efficient management with hemostatic procedures, such as bimanual compression of the uterus, intrauterine gauze packing, balloon tamponade, and DIC treatment, is necessary [12]. Currently available DIC treatments consist of blood product transfusion; tranexamic acid; and anticoagulants such as antithrombin III (AT III), protease inhibitors, and thrombomodulin [18-20]. Unfractionated heparin (UFH) and low molecular weight heparin (LMWH) are also sometimes used in obstetric DIC. However, their risks of causing critical bleeding adverse events during childbirth are not yet enough understood, and the evidence for which of the heparins (UFH versus LMWH) is safer during childbirth is currently lacking [1]. Compared to non-obstetrical DIC, such as cancer-induced DIC, obstetric DIC is more likely to present with critical bleeding based on consumption coagulopathy rather than procoagulant form [1,21]. Therefore, evidence is needed regarding the optimal choice of anticoagulant in peripartum women. To achieve this, the present study investigated a Japanese nationwide administrative database with a large number of women with childbirth, and the risk of critical obstetrical bleeding with each type of anticoagulant was compared.

The article "Risk Assessment of Critical Obstetric Bleeding With Low-Molecular-Weight Heparin" was published in 2024. Journal: Cureus.

## Materials and methods

Study design and population

The present study retrospectively investigated the Japanese Diagnosis Procedure Combination (DPC) database, which covers approximately 70% of the annual hospitalization episodes in Japan. The study was conducted from April 2018 to March 2022. Because the present study aimed to investigate the risk of critical obstetric bleeding with each obstetric condition and anticoagulation among women during childbirth, hospitalization episodes without childbirth were not collected. Furthermore, women who gave birth but had an uncertain date of childbirth were excluded in order to focus on the risk factors of critical bleeding during childbirth. Data regarding the used treatment profiles and outcomes of DIC represented by (1) all-cause mortality, (2) total hysterectomy, and (3) massive red blood cell (RBC) transfusion, were comprehensively collected. The obstetric and therapeutic risk factors for the development of critical obstetric bleeding were first investigated among the overall women with childbirth. Then, the obstetric and therapeutic risk factors of critical obstetric bleeding were further investigated among the women with obstetrical DIC. A flow diagram of the study design is shown in Figure 1.

**Figure 1:** Flow diagram of the study design Initial data from 2018–2022 collected from all Diagnosis Procedure Combination (DPC) hospitals included more than 30 million hospitalization episodes. From this data, information from those without childbirth or with an uncertain delivery date was excluded. From the remaining women with a certain date of childbirth during the study period, those who developed obstetric DIC were selected for the subsequent analyses of treatment profiles and the prognostic impact of each treatment. AT III: antithrombin III; DIC: disseminated intravascular coagulation; FFP: fresh frozen plasma; LMWH: low-molecular-weight heparin; RBC: red blood cell; UFH: unfractionated heparin The figure was drawn by the authors of this article.

Evaluated variables

The variables evaluated among women with obstetric DIC included age at hospitalization with childbirth, obstetrical background, use of blood product transfusion and intravenously administered anticoagulation therapies, and outcomes of obstetric DIC. The evaluated obstetrical backgrounds included the type of childbirth (vaginal, elective cesarean section (CS), and emergent CS), placental abruption, amniotic embolism, low-lying placenta (LLP)/placenta previa (PP), placenta accreta spectrum, uterine rupture, eclampsia, hemolysis, elevated liver enzymes and low platelet (HELLP) syndrome, atonic bleeding, uterine inversion, and birth canal laceration. The evaluated blood products included RBC, platelets, and fresh frozen plasma (FFP) transfusions. The intravenous anticoagulation therapies evaluated included UFH, LMWH, AT III, protease inhibitors, and thrombomodulin. In addition to these anticoagulants, the use of protamine to reverse the heparin activity and intravenous tranexamic acid were further investigated. The DIC outcome was defined as the subsequent occurrence of death, total hysterectomy, or massive RBC transfusion.

The article "Risk Assessment of Critical Obstetric Bleeding With Low-Molecular-Weight Heparin" was published in 2024. Journal: Cureus.

Statistical analysis

Distributions of the quantitative data are reported as the median and interquartile range (IQR; 25-75 percentiles). Comparisons of quantitative data between the two groups were performed using the Mann-Whitney U test. The effect size r was reported together with the p-value. Qualitative data were compared between the two groups using the chi-square test or Fisher’s exact test, according to the expected frequency of each subgroup. Unadjusted odds ratio (OR) was reported as the effect size together with a 95% confidence interval (CI). To investigate the relationship between an outcome and one or more explanatory variables, including data with complete separation, Firth’s logistic regression analysis based on a penalized likelihood method was performed using either total hysterectomy or massive RBC transfusion as the dependent variable [22]. For both outcomes, all explanatory variables of interest were simultaneously entered into the respective regression models, and the risk of multicollinearity between the explanatory variables was evaluated by calculating the variance inflation factor (VIF) for each variable. Adjusted OR (aOR) and 95% CI are reported. A massive RBC transfusion was defined as a daily transfusion of ≥ 4,000 cc, as the mortality rate become greater than 1.0% using this cutoff [23]. Logistic regression analysis was not performed for the outcome of death because the number of women with this outcome was not large enough. Multiple linear regression analyses were further performed to evaluate the independent impact of the evaluated anticoagulants on the blood loss amount during childbirth by using the administrations of UFH, LMWH, AT III, protease inhibitor, and thrombomodulin as the explanatory variables. Two-sided p-values <0.05 were considered statistically significant, and the alpha level was not adjusted for multiple comparisons based on the exploratory and descriptive nature of the present study [24]. R, version 4.1.3 statistical software (R Foundation for Statistical Computing, Vienna, Austria) and JMP Pro 17 (SAS Institute Inc., Cary, NC, USA) were used for analyses.

Ethics

This study was approved by the Institutional Review Boards of Tokyo Medical and Dental University (approval number: M2000-788) and Tohoku University Graduate School of Medicine (approval number: 2022-1-441). The review board waived the requirement for written informed consent because patient data were anonymous. All procedures in this study were conducted in accordance with the latest version of the Declaration of Helsinki, as revised in 2013.

## Results

Overall population of women with childbirth

Of the 30,557,174 hospitalization episodes occurring during the study period, 354,299 were with certain dates of childbirth during the period. The median age of the 354,299 women was 33 (IQR 30-37) years. Among the overall 354,299 women with childbirth, the number of women treated with each of the following treatments during the peripartum period was as follows: RBC transfusion in 10,119 (2.9%), platelet transfusion in 1,917 (0.5%), FFP transfusion in 6,389 (1.8%), UFH in 62,084 (17.5%), LMWH in 1,986 (0.6%), AT III in 2,769 (0.8%), protease inhibitors in 1,241 (0.4%), and thrombomodulin in 168 women (0.05%). The median of the administered daily dose of UFH on the day of childbirth was 5,000 units (IQR 5,000-8,333 units), and the same of LMWH was 5,000 units (IQR 5,000-5,000 units). There were 142 women (0.04%) who were treated by both UFH and LMWH. Protamine to reverse the heparin activity was used in 109 women (0.03%). Intravenous tranexamic acid was used in 19,944 women (5.6%). The number of women with each of the following non-obstetrical and obstetrical complications was as follows: pulmonary embolism in 215 (0.06%), deep-vein thrombosis in 1,808 (0.5%), hypertension in 4,034 (1.1%), diabetes mellitus in 4,489 (1.3%), iron-deficiency anemia in 56,321 (15.9%), obstetrical DIC in 3,099 (0.9%), amniotic embolism in 79 (0.02%), HELLP syndrome in 1,577 (0.4%), placental abruption in 4,116 (1.2%), LLP/PP in 15,477 (4.4%), and atonic bleeding in 40,725 women (11.5%).

The article "Risk Assessment of Critical Obstetric Bleeding With Low-Molecular-Weight Heparin" was published in 2024. Journal: Cureus.

As major obstetric outcomes, maternal death occurred in 38 (0.01%), and massive RBC transfusion ≥4,000 cc was administered in 484 women (0.1%). The crude and adjusted ORs for the requirement of massive RBC transfusion ≥4,000 cc among the overall 354,299 women by the types of anticoagulants are listed in the upper half of Table 1. Among the evaluated five types of anticoagulation treatments, only the LMWH showed no significant association with the subsequent massive RBC transfusion in both univariate (OR, 0.74; 95% CI, 0.09-2.68) and multivariable analyses (aOR, 0.54; 95% CI, 0.11-2.71). A subgroup analysis among the 274,568 women with elective or emergent CS was further performed (lower half of Table 1). Again, all evaluated anticoagulants were significantly associated with a higher incidence of critical bleeding, only except for LMWH. As another major obstetric outcome, total hysterectomy was performed in 180 women (0.05%), including 68 with obstetrical DIC. The most common obstetrical background was atonic bleeding (n=87), followed by placenta accreta spectrum (n=82) and LLP/PP (n=72). Of them, 37 were with overlapping LLP/PP and placenta accreta spectrum.

**Table 1:** Factors related to massive RBC transfusion among the overall 354,299 women with childbirth Unadjusted and adjusted OR for the requirement of massive RBC transfusion ≥ 4,000 cc were calculated among the overall 354,299 women for each obstetrical condition. Adjusted ORs were calculated with the binary logistic regression analysis by simultaneously entering all explanatory variables into the model. OR: odds ratio; RBC: red blood cell; VIF: variance inflation factor; LMWH: low-molecular-weight heparin; AT III, antithrombin III; DIC, disseminated intravascular coagulation; UFH, unfractionated heparin; CS: cesarean section *Adjusted ORs and 95% CI were obtained by performing a multiple logistic regression analysis

Characteristics	Unadjusted Results		Adjusted Results		VIF
	OR (95% CI)	P-value	OR (95% CI)	P-value	
Population: overall 354,299 women					
Age per 1 year	1.08 (1.06 – 1.10)	<0.001	1.07 (1.05 – 1.09)	<0.001	1.018
Vaginal delivery	1.00 (reference)	–	1.00 (reference)	–	–
Elective CS	0.34 (0.27 – 0.44)	<0.001	0.24 (0.18 – 0.32)	<0.001	1.164
Emergent CS	0.85 (0.70 – 1.05)	0.128	0.28 (0.22 – 0.36)	<0.001	1.169
Obstetrical DIC	230.63 (190.71 – 278.91)	<0.001	52.22 (40.44 – 67.41)	<0.001	1.233
UFH	25.66 (19.97 – 33.34)	<0.001	17.91 (13.71 – 23.40)	<0.001	1.063
LMWH	0.74 (0.09 – 2.68)	0.665	0.54 (0.11 – 2.71)	0.455	1.004
AT III	81.81 (67.36 – 99.08)	<0.001	2.61 (2.01 – 3.38)	<0.001	1.196
Protease inhibitors	49.99 (37.96 – 65.07)	<0.001	1.72 (1.22 – 2.41)	0.002	1.044
Thrombomodulin	257.68 (173.58 – 377.54)	<0.001	5.19 (3.26 – 8.26)	<0.001	1.040
Population: 274,568 women with elective or emergent CS					
Age per 1 year	1.06 (1.04 – 1.09)	<0.001	1.06 (1.04 – 1.08)	<0.001	1.010
Elective CS	1.00 (reference)	–	1.00 (reference)	–	–
Emergent CS	2.50 (1.98 – 3.15)	<0.001	1.17 (0.90 – 1.15)	0.235	1.015
Obstetrical DIC	174.61 (139.34 – 218.81)	<0.001	50.46 (37.17 – 68.50)	<0.001	1.216
UFH	21.18 (15.49 – 28.94)	<0.001	13.06 (9.48 – 18.00)	<0.001	1.009
LMWH	0.43 (0.06 – 3.06)	0.399	0.22 (0.03 – 1.93)	0.172	1.002
AT III	70.95 (56.28 – 89.44)	<0.001	2.74 (1.99 – 3.76)	<0.001	1.178
Protease inhibitors	45.92 (33.59 – 62.78)	<0.001	1.85 (1.25 – 2.71)	0.002	1.039
Thrombomodulin	254.31 (163.68 – 395.12)	<0.001	4.88 (2.84 – 8.38)	<0.001	1.039

Factors associated with obstetrical DIC

A total of 3,099 women were diagnosed with obstetrical DIC. Those with DIC and without the registered diagnosis of “obstetrical DIC” were not counted to reduce the population heterogeneity. The median age of the 3,099 women was 34 (IQR 30-38) years, which was higher than that of women without obstetrical DIC (33 (IQR 30-37) years; effect size r = 0.01, p<0.001). Of the 3,099 women, 13 (0.4%) died during childbirth. Of the 3,099 women, 68 (2.2%) underwent total hysterectomy, including two died during childbirth. Pulmonary embolism was seen in 18 (0.6%; two died), and deep-vein thrombosis was seen in 37 women (1.2%; none died). These rates were significantly higher than those in the other 351,200 non-DIC women (0.06% and 0.5%, respectively; p<0.001 for both). Obstetrical and non-obstetrical conditions potentially associated with the development of obstetrical DIC are summarized in Table 2. The most common obstetrical complication was atonic bleeding (n=1,300; 41.9%), followed by placental abruption (n=362; 11.7%), LLP/PP (n=264; 8.5%), and placenta accreta spectrum (n=218; 7.0%). The calculated crude OR was the highest for amniotic embolism (OR, 301.48; 95% CI, 179.21-508.05), followed by uterine inversion (OR, 44.65; 95% CI, 29.61-66.01).

The article "Risk Assessment of Critical Obstetric Bleeding With Low-Molecular-Weight Heparin" was published in 2024. Journal: Cureus.

**Table 2:** Obstetrical and non-obstetrical factors in relation to obstetrical DIC As prior non-obstetrical conditions before childbirth that are potentially associated with obstetrical DIC, IDA, ITP, SLE, and APS were evaluated. The odds ratios were calculated among the overall 354,299 women. APS: antiphospholipid antibody syndrome; CI: confidence interval; CS: cesarean section; DIC: disseminated intravascular coagulation; HELLP: hemolysis, elevated liver enzymes and low platelets; IDA: iron-deficiency anemia; ITP: idiopathic thrombocytopenic purpura; LLP: low-lying placenta; OR: odds ratio; PP: placenta previa; SLE: systemic lupus erythematosus *Percentages were calculated among those with or without the obstetric characteristics.

Obstetrical factors	n	Obstetrical DIC, n (%)*		OR (95% CI)	P-value
		Among those with each factor	Among those without each factor		
Vaginal childbirth	79,731	766 (1.0 %)	2,333 (0.9 %)	1.13 (1.04 – 1.23)	0.003
Elective CS	151,403	517 (0.3 %)	2,582 (1.3 %)	0.27 (0.24 – 0.29)	<0.001
Emergent CS	123,165	1,816 (1.5 %)	1,283 (0.6 %)	2.68 (2.49 – 2.88)	<0.001
Placental abruption	4,116	362 (8.8 %)	2,737 (0.8 %)	12.24 (10.92 – 13.72)	<0.001
Amniotic embolism	79	57 (72.2 %)	3,042 (0.9 %)	301.48 (179.21 – 508.05)	<0.001
LLP and PP	15,477	264 (1.7 %)	2,835 (0.8 %)	2.06 (1.80 – 2.34)	<0.001
Placenta accreta	3,175	218 (6.9 %)	2,881 (0.8 %)	8.91 (7.69 – 10.28)	<0.001
Uterine rupture	230	25 (10.9 %)	3,074 (0.9 %)	13.93 (8.79 – 21.18)	<0.001
Eclampsia	738	37 (5.0 %)	3,062 (0.9 %)	6.04 (4.21 – 8.43)	<0.001
HELLP	1,577	159 (10.1 %)	2,940 (0.8 %)	13.34 (11.21 – 15.79)	<0.001
Atonic bleeding	40,725	1,300 (3.2 %)	1,799 (0.6 %)	5.71 (5.31 – 6.14)	<0.001
Uterine inversion	132	37 (28.0 %)	3,062 (0.9 %)	44.65 (29.61 – 66.01)	<0.001
Birth canal laceration	8,937	120 (1.3 %)	2,979 (0.9 %)	1.56 (1.29 – 1.88)	<0.001
IDA	56,321	613 (1.1%)	2,486 (0.8%)	1.31 (1.19 – 1.43)	<0.001
ITP	345	5 (1.4%)	3,094 (0.9%)	1.67 (0.54 – 3.93)	0.235
SLE	728	13 (1.8%)	3,086 (0.9%)	2.06 (1.09 – 3.56)	0.015
APS	557	9 (1.6%)	3,090 (0.9%)	1.86 (0.85 – 3.57)	0.067

Regarding the intravenously administered treatments, 2,289 (73.9%) were treated with RBC transfusion, 786 (25.4%) with platelet transfusion, 2,262 (73.0%) with FFP transfusion, 1,354 (43.7%) with UFH, 29 (0.9%) with LMWH, 1,162 (37.5%) with AT III, 368 (11.9%) with protease inhibitor, and 133 (4.3%) with thrombomodulin. Among the 3,099 women, the median of the administered daily dose of UFH on the day of childbirth was 5,000 units (IQR 5,000-10,000 units), and the same of LMWH was 5,000 units (IQR 4,000-5,000 units). To investigate the effect of each DIC treatment on the two primary study outcomes (maternal death and total hysterectomy), univariate analysis was performed for each type of treatment (Table 3). For the mortality (upper half of Table 3), UFH (OR, 4.32; 95% CI, 1.11-24.47) was with a significant OR greater than 1.0, while LMWH was not (OR, 3.84; 95% CI, 0.03-30.15). For the requirement of total hysterectomy (lower half of Table 3), UFH was with a significant OR greater than 1.0 (OR, 4.31; 95% CI, 2.41-8.13), while LMWH was not (OR, 0.74; 95% CI, 0.01-5.38).

The article "Risk Assessment of Critical Obstetric Bleeding With Low-Molecular-Weight Heparin" was published in 2024. Journal: Cureus.

**Table 3:** Maternal death and total hysterectomy by the administered DIC treatments among the 3,099 women with obstetrical DIC AT III: antithrombin III; CI: confidence interval; DIC: disseminated intravascular coagulation; FFP: fresh frozen plasma; LMWH: low-molecular-weight heparin; OR: odds ratio; RBC: red blood cell; UFH: unfractionated heparin *Firth’s logistic regression analysis for variables with complete separation

Treatments	Maternal Death, n (%)		Crude OR (95% CI)	P-value
	Among those with each treatment	Among those without each treatment		
Total hysterectomy (n=68)	2 (2.9%)	11 (0.4%)	8.32 (1.81 – 38.28)	0.032
RBC transfusion (n=2,289)	11 (0.5%)	2 (0.3%)	1.95 (0.42 – 18.15)	0.534
Platelet transfusion (n=786)	10 (1.3%)	3 (0.1%)	9.91 (2.54 – 56.20)	<0.001
FFP transfusion (n=2,262)	11 (0.5%)	2 (0.2%)	2.04 (0.44 – 18.98)	0.534
UFH (n=1,354)	10 (0.7%)	3 (0.2%)	4.32 (1.11 – 24.47)	0.022
LMWH (n=29)*	0 (0.0%)	13 (0.4%)	3.84 (0.03 – 30.15)	0.442
AT III (n=1,162)	4 (0.3%)	9 (0.5%)	0.74 (0.17 – 2.66)	0.777
Protease inhibitors (n=368)	4 (1.1%)	9 (0.3%)	3.32 (0.74 – 11.98)	0.059
Thrombomodulin (n=133)	2 (1.5%)	11 (0.4%)	4.10 (0.44 – 19.06)	0.105
Treatments	Total hysterectomy, n (%)		Crude OR (95% CI)	P-value
	Among those with each treatment	Among those without each treatment		
RBC transfusion (n=2,289)	66 (2.9%)	2 (0.3%)	11.99 (3.18 – 101.34)	<0.001
Platelet transfusion (n=786)	51 (6.5%)	17 (0.7%)	9.36 (5.28 – 17.41)	<0.001
FFP transfusion (n=2,262)	67 (3.0%)	1 (0.1%)	25.51 (4.41 – 1,019.43)	<0.001
UFH (n=1,354)	52 (3.8%)	16 (0.9%)	4.31 (2.41 – 8.13)	<0.001
LMWH (n=29)*	0 (0.0%)	68 (2.2%)	0.74 (0.01 – 5.38)	0.828
AT III (n=1,162)	28 (2.4%)	40 (2.1%)	1.17 (0.67 – 1.96)	0.612
Protease inhibitors (n=368)	7 (1.9%)	61 (2.2%)	0.849 (0.33 – 1.88)	0.850
Thrombomodulin (n=133)	8 (6.0%)	60 (2.0%)	3.10 (1.25 – 6.69)	0.008

Logistic regression analyses for major outcomes in obstetrical DIC

To adjust for the effects of simultaneously administered DIC treatments on outcomes represented by the requirements of total hysterectomy (n=68), massive RBC transfusion ≥ 4,000 cc (n=313), and major obstetric hemorrhage with childbirth-related blood loss ≥ 1,500 cc (n=1,465) among the 3,099 women with obstetrical DIC, logistic regression analysis was performed for each outcome (Figure 2). To deal with the bias caused by the separation problem, Firth’s logistic regression analyses were performed for the two outcomes of total hysterectomy and massive RBC transfusion. Age, platelet transfusion, UFH, LMWH, AT III, protease inhibitor, and thrombomodulin levels were used as independent variables. RBC and FFP transfusions were not included in this first model to avoid the risk of multicollinearity. For the requirement of total hysterectomy (top of the panel), higher ages, platelet transfusion, UFH, and thrombomodulin were with significant aORs greater than 1.0, while LMWH was not. For the requirement of massive RBC transfusion (middle of the panel), higher ages, platelet transfusion, UFH, AT III, and thrombomodulin were with significant aORs greater than 1.0, while LMWH was not. For the occurrence of major obstetric hemorrhage with childbirth-related blood loss ≥ 1,500 cc, higher ages, platelet transfusion, UFH, and AT III were with significant aORs greater than 1.0, while LMWH was not.

The article "Risk Assessment of Critical Obstetric Bleeding With Low-Molecular-Weight Heparin" was published in 2024. Journal: Cureus.

**Figure 2:** Logistic regression analyses for hysterectomy, RBC transfusion ≥4,000 cc, and blood loss during childbirth ≥1,500 cc Data from 3,099 women with obstetrical DIC were used. Firth’s logistic regression analysis was performed with the two outcomes of total hysterectomy and massive RBC transfusion to reduce the bias caused by separation. Data on DIC severity and pathological form were not available; therefore, they were substituted by the history of platelet transfusion. Error bars represent 95% confidence intervals for the adjusted ORs. AT III: antithrombin III; CI: confidence interval; DIC: disseminated intravascular coagulation; LMWH: low-molecular-weight heparin; OR: odds ratio; UFH: unfractionated heparin; VIF: variance inflation factor The figure was drawn by the authors of this article.

Heparin and the total amount of RBC transfusion

Based on the finding that the use of UFH was associated with massive RBC transfusion in obstetrical DIC, the Spearman’s correlation coefficient between the administered daily dose of UFH or LMWH on the day of childbirth and the total RBC transfusion was calculated among the 3,099 women with obstetrical DIC. A significant positive correlation was confirmed between the daily dose of UFH on the day of childbirth and the total RBC transfusion amount (Spearman’s ρ=0.293; p<0.001), whereas it was absent between the daily dose of LMWH on the day of childbirth and RBC transfusion amount (ρ=−0.048; p=0.008). The significant positive correlation with the daily dose of UFH was reproduced when the same analysis was performed on those who were treated by UFH on the day of childbirth (ρ=0.171; p<0.001), suggesting a dose-dependent effect of UFH to the obstetrical hemorrhage.

To check that the significant association between the dose of UFH and RBC transfusion amount was irrespective of the other relevant confounders (age, delivery type, protamine, intravenous tranexamic acid), a multiple linear regression analysis for the total amount of RBC transfusion was performed by simultaneously entering the following six explanatory variables: age, delivery type, dose of UFH on the day of childbirth, dose of LMWH on the day of childbirth, the use of protamine to reverse the heparin activity, and the use of intravenous tranexamic acid. As a result, the dose of UFH on the day of childbirth was significantly associated with the total RBC transfusion amount (standardized coefficient β=0.271, p<0.001), whereas the dose of LMWH was not (β=−0.022, p=0.171).

## Discussion

The present study demonstrated that the use of LMWH was not associated with a higher incidence of critical obstetric bleeding both in the overall women with childbirth and in those with obstetrical DIC. Meanwhile, the use of UFH was associated with a higher incidence of critical obstetric bleeding. Another notable finding was that nearly half of the women with obstetric DIC were treated by UFH in Japan. One of the reasons may be the empirical use of UFH for women suspected of amniotic fluid embolism [25-27], although its effectiveness remains controversial. Another notable finding was that a higher maternal age was associated with higher risks of obstetric DIC, critical bleeding, and total hysterectomy. Total hysterectomy is an effective hemostatic procedure to save maternal life, but it is better to avoid in view of fertility preservation. The overall incidence of total hysterectomy in this study was 0.51 per 1,000 deliveries, which was almost consistent with a previous study from Romania with 0.99 per 1,000 deliveries [28]. Currently, the marriage and childbirth ages both continue to gradually increase in many developed countries, suggesting increased risks of critical obstetric bleeding. Choosing LMWH instead of UFH to use during childbirth will hopefully contribute to avoiding hysterectomy.

The article "Risk Assessment of Critical Obstetric Bleeding With Low-Molecular-Weight Heparin" was published in 2024. Journal: Cureus.

The observed frequency of obstetrical DIC among the initially recruited 354,299 women with childbirth was 0.9 % (n=3,099); however, this rate could be unreliable as most of the women who delivered without any complications, including DIC, were not included in the DPC database [29]. Considering that the annual number of childbirths in Japan is approximately 800,000, the total number of childbirths in Japan during the study period would be approximately 3 to 4 million. Because the majority of women with obstetrical DIC are typically transferred to a DPC hospital, the actual prevalence of obstetrical DIC in Japan can be estimated to be approximately 0.1%, which falls within the worldwide expected prevalence [1].

Currently available anticoagulants for DIC treatment include UFH, LMWH, AT III, synthetic protease inhibitors, and recombinant human thrombomodulin. Heparin exerts anticoagulant activity in an AT-dependent manner with its affinity for AT III [30]. In contrast to this, synthetic serine protease inhibitors (nafamostat mesilate, gabexate mesilate) exert anticoagulant activity in an AT-independent manner, and they are known to be with low risks of major hemorrhagic side effects [31,32]. Recombinant thrombomodulin is a relatively new DIC treatment with both anticoagulant and anti-inflammatory effects [33]. This agent could be a good choice for patients with DIC accompanied by conditions presenting systemic inflammation, such as sepsis [21]. There is only limited evidence for recombinant thrombomodulin in obstetric DIC, and its use for obstetric DIC is currently limited to those with insufficient anticoagulant effects by other anticoagulation therapies. Whether recombinant thrombomodulin can be used as a first-line anticoagulant in obstetric DIC still remains undetermined, and further studies are needed after stratifying the causative obstetric disorders [34]. This study showed significant crude ORs and aORs with the use of thrombomodulin for the subsequent requirement of total hysterectomy and massive RBC transfusion, but these findings require cautious interpretations. Since the approval of the drug for treating DIC in Japan in 2008, its indication for obstetric DIC still remains inconclusive. Currently, the use of thrombomodulin in obstetric DIC is limited to situations where the benefits are expected to exceed the risks, and it is used for cases in which other anticoagulants are ineffective. Therefore, women treated with thrombomodulin in the present study might have had more severe DIC at baseline. Consequently, it remains uncertain whether the findings of the present study truly indicated the risk of using thrombomodulin for obstetric DIC. A previous study reported that thrombomodulin may improve clinical and laboratory findings, such as platelet counts, D-dimer levels, and fibrinogen levels in obstetric DIC [34,35]. Further studies are needed to confirm the benefits and safety of using thrombomodulin in obstetric DIC.

The article "Risk Assessment of Critical Obstetric Bleeding With Low-Molecular-Weight Heparin" was published in 2024. Journal: Cureus.

This study had several limitations. First, the DIC score for each individual was unavailable in the nationwide DPC database. Therefore, the analyses could not be adjusted for baseline clinical severity and laboratory findings in women with obstetric DIC. Similarly, whether each patient had a procoagulant, predominantly with thrombotic complications, or a hyperfibrinolytic form of DIC with bleeding complications could not be identified from the database. Moreover, this study did not evaluate the subsequent organ dysfunction due to DIC. The results of the present study certainly imply that UFH increases the risk of major obstetrical bleeding and subsequently total hysterectomy and mortality; however, this may not necessarily indicate that UFH is hazardous and should be avoided in all women with obstetrical DIC. Heparin may be beneficial in cases of hypercoagulation. Using LMWH rather than UFH may decrease the risk of negative outcomes. A meta-analysis suggested that the risk of heparin-induced thrombocytopenia is lower with LMWH than with UFH [36]. The clinical and laboratory findings of women with obstetric DIC should be assessed to correctly interpret the risk of thrombotic organ dysfunction with hypercoagulation before deciding on the use of heparin in each case. Another limitation of this study is that it could not statistically investigate the hemostatic effect of intravenous tranexamic acid in obstetric DIC because of its retrospective nature [19]. In a recent randomized, double-blind, placebo-controlled WOMAN trial, women with obstetrical DIC who received 1 g of intravenous tranexamic acid in addition to usual care showed a lower mortality rate due to bleeding than those who received the placebo, especially in those who were administered tranexamic acid within 3 h of delivery [37]. Fibrinogen concentrate is another promising option for treating DIC, which was not evaluated in this study. As a large amount of FFP transfusion may cause pulmonary edema, fibrinogen concentrate would be helpful to reduce the required FFP transfusion amount and avoid the side effects [38].

The article "Risk Assessment of Critical Obstetric Bleeding With Low-Molecular-Weight Heparin" was published in 2024. Journal: Cureus.

## Conclusions

The use of UFH was associated with an increased rate of negative outcomes derived from uncontrollable massive obstetrical hemorrhage, while the use of LMWH was not. The findings suggested that an administration of UFH should be carefully decided considering the estimated hypercoagulative status in each patient. LMWH would be safer than UFH in women during childbirth. Future prospective studies to determine the risk of using UFH and the safety of LMWH during childbirth are warranted.
